The article "Estimation of Gait Parameters for Transfemoral Amputees Using Lower Limb Kinematics and Deterministic Algorithms" was published in 2022. Journal: Appl Bionics Biomech.

# Estimation of Gait Parameters for Transfemoral Amputees Using Lower Limb Kinematics and Deterministic Algorithms

**DOI:** 10.1155/2022/2883026

**Published:** 2022-10-19

**Authors:** Zohaib Aftab, Gulraiz Ahmed, Asad Ali, Nazia Gillani

**Affiliations:** ^1^Faculty of Engineering, University of Central Punjab, Lahore 54000, Pakistan; ^2^Human-Centered Robotics Lab, National Center of Robotics and Automation, University of Central Punjab, Lahore, Pakistan; ^3^School of Engineering, University of Edinburgh, Edinburgh, UK

## Abstract

Accurate estimation of gait parameters depends on the prediction of key gait events of heel strike (HS) and toe-off (TO). Kinematics-based gait event estimation has shown potential in this regard, particularly using leg and foot velocity signals and gyroscopic sensors. However, existing algorithms demonstrate a varying degree of accuracy for different populations. Moreover, the literature lacks evidence for their validity for the amputee population. The purpose of this study is to evaluate this paradigm to predict TO and HS instants and to propose a new algorithm for gait parameter estimation for the amputee population. An open data set containing marker data of 12 subjects with unilateral transfemoral amputation during treadmill walking was used, containing around 3400 gait cycles. Five deterministic algorithms detecting the landmarks (maxima, minima, and zero-crossings [ZC]) in the foot, shank, and thigh angular velocity data indicating HS and TO events were implemented and their results compared against the reference data. Two algorithms based on foot and shank velocity minima performed exceptionally well for the HS prediction, with median accuracy in the range of 6–13 ms. However, both these algorithms produced inferior accuracy for the TO event with consistent early prediction. The peak in the thigh velocity produced the best result for the TO prediction with <25 ms median error. By combining the HS prediction using shank velocity and TO prediction from the thigh velocity, the algorithm produced the best results for temporal gait parameters (step, stride times, stance, and double support timings) with a median error of less than 25 ms. In conclusion, combined shank and thigh velocity-based prediction leads to improved gait parameter estimation than traditional algorithms for the amputee population.

## 1. Introduction

Gait analysis is a valuable tool in assessing various pathologies as well as in quantifying outcomes of an intervention. A pre-requisite to effective gait analysis is the identification of key gait events of heel strike (HS) and toe-off (TO), which represent the moments the foot is placed and removed from the ground, respectively [1]. Incorrect gait event detection leads to inaccurate gait segmentation into stance and swing phases, leading to erroneous spatio-temporal parameters. Moreover, it is also important for objective evaluation of clinical outcomes for amputees [2].

The article "Estimation of Gait Parameters for Transfemoral Amputees Using Lower Limb Kinematics and Deterministic Algorithms" was published in 2022. Journal: Appl Bionics Biomech.

The gold standard for event prediction is the ground reaction force (GRF) obtained from specialized force platforms in research laboratories. However, due to high cost and space constraints, this method is limited to research studies. Moreover, it only detects events from a limited number of steps (usually one or two) depending upon the number of force platforms.

In the absence of reliable force data, algorithm-based event detection methods using optoelectronic (marker) data [4], [5] or inertial sensors are exploited. These methods rely on leg or foot kinematics and rule-based algorithms to estimate gait events. Many authors have validated this approach for healthy subjects [5]–[12] as well as for subjects with gait disorders [3], [13]–[16] with varying degrees of accuracy.

The kinematic methods require an algorithm to identify observable features in the velocity/acceleration data of body segments. Several rule-based algorithms have also been developed for this purpose. A popular choice is to use the shank angular velocity for TO and HS estimation corresponding to the minima in the sagittal plane angular velocity signal [17]. Many researchers have exploited this signal over the years for diverse subject populations [5], [6], [10], [15], [18]–[22]. Though reasonable accuracy may be achieved for the HS event (errors of less than 10 ms), its validity for the TO event has been subject to some debate. Larger discrepancies (of the order of 80 ms) were reported for TO prediction using this algorithm by some studies [23], [24], questioning its validity for different populations. Other studies have explored the potential of the ZC point of the signal to predict gait events and have shown better results for certain populations [10], [16].

Although less frequently done, shank and foot acceleration-based algorithms have also been exploited by some researchers. However, it has been shown that acceleration-based methods frequently present larger errors [25] or contain multiple false positives which are difficult to distinguish automatically (see discussion in [3]). Other studies have advocated foot angular velocity be a better predictor of gait events than shank velocity [12], [26]. In all, there is little consensus among researchers regarding the best kinematic approach for automatic event detection, especially for the TO event.

Even lesser evidence is available for the validity of this approach for the amputee gait. Since lower-body amputations lead to gait deviations and compensatory movements, existing kinematic methods may render erroneous results. Only a handful of studies have focused on the amputee population [27]–[30]. Researchers in [27] experimented with only one amputee subject hence limiting the generalization of their results. Bastas and colleagues included a group of 16 transfemoral (TF) amputees but only used single Inertial Measurement Unit data mounted in the lower-back region [28]. Researchers in [30] presented a threshold-based algorithm using state machines for real-time detection. The algorithm required training data for optimized threshold calculation and constraining windows increasing its complexity and computational cost. Lastly, authors in [29] included seven TF amputees with a unilateral amputation using a microprocessor-controlled knee. They explored several velocity and acceleration-based algorithms and obtained the best results with the one proposed by Trojaniello and colleagues [31]. However, the algorithm lacked accuracy when predicting some gait parameters including the double support duration.

The article "Estimation of Gait Parameters for Transfemoral Amputees Using Lower Limb Kinematics and Deterministic Algorithms" was published in 2022. Journal: Appl Bionics Biomech.

This study aims to compare the accuracy of some existing kinematic algorithms in predicting gait events for the amputee population and propose a novel algorithm to improve the accuracy of the temporal gait parameters. It extends the previously published preliminary study by authors [32], [33]. As demonstrated in the next sections, the new algorithm greatly improves the accuracy of the TO event resulting in improved gait parameter estimation at all speeds. The velocity of the foot and leg segments is calculated from the marker data while the validation is done against the force platform data.

This article is structured as follows: Section 2 details the data set used in this study as well as the working of algorithms. Results are presented in Section 3, while Section 4 concludes the article.

## 2. Materials and Methods

### 2.1. Data Set

In order to test various algorithms, a data set of 18 individuals with unilateral TF amputation from [34] is used. All individuals in this study had a unilateral above-knee amputation for at least one year. The participants wore the prescribed prosthesis for a minimum of six months using it at least three hours daily. These subjects and their data are presented in Table 1. All individuals were inquired about their experiences in the past of using a treadmill for walking. Training was provided to individuals who had little or no experience using a treadmill with a prosthesis.

It is the most comprehensive data set of prosthesis users which provides force platform data for all steps taken during a trial. According to the subjects' preferred walking speed and dependency on the handrails, the subjects were split into two groups. On the Medicare functional categorization level, they were classified as either K-level 2 or K-level 3. A person was placed in the K2 group if they needed handrails to walk at any speed more than 0.8 m/s or if their top walking speed was 0.8 m/s. This group of subjects walked at five different speeds of [0.4, 0.5, 0.6, 0.7, and 0.8 m/s]. Similarly, if subjects could walk at speeds up to 1.2 m/s without using handrails, they were assigned to the K3 group, and they walked at speeds of [0.6, 0.8, 1.0, 1.2, and 1.4 m/s].

The article "Estimation of Gait Parameters for Transfemoral Amputees Using Lower Limb Kinematics and Deterministic Algorithms" was published in 2022. Journal: Appl Bionics Biomech.

The original study contained an equal number of subjects in both groups. However, for this study, subjects/trials using the handrails during walking were excluded. This allowed a uniform protocol across all subjects for objective inter-subject comparison. As a result, 270 walking trials from 12 subjects were available for further analysis (including three K-level 2 and nine K-level 3 subjects).

### 2.2. Estimation of Angular Velocity Signal from Marker Data

The raw data consisted of 61 cutaneous reflective markers' three-dimensional trajectories. The data contained the .c3d files for the marker trajectories which were retrieved using an open-source motion analyzer software Motion Kinematic and Kinetic Analyzer [35]). The data for each trial was exported to a .csv file and read in MATLAB to calculate angular velocities from marker coordinates. Shank and thigh velocities were calculated using two markers in line with the bone axis (TIB and TIBI for shank, and THI and THII for thigh, Figure 1) using the method described in [36]. Foot velocity was calculated using heel and toe markers (marked HEE and TOE, respectively).

The raw marker data was collected at 200 Hz and it is subject to a lot of noise due to soft tissue artifacts. To reduce the noise in the resulting angular velocity signal, a low pass filter was designed and implemented. For this purpose, the frequency spectrum and the Nyquist frequency of the signal for all subjects were analyzed. A cut-off frequency of 4 Hz wave was chosen which resulted in negligible loss of data and time-shift of the signal.

### 2.3. Algorithms

A total of five algorithms based on the sagittal plane angular velocities of three segments (foot, shank, and thigh) are developed in MATLAB. Representative velocity signals, calculated from the reflexive marker data (detailed in the next section), are shown in Figure 1.

For the foot and shank velocities, a dual-minima (DM) algorithm similar to the one presented in [22] is implemented (termed S-DM and F-DM algorithms). It starts with the detection of all the positive peaks (maxima) of the signal. These positive peaks are associated with the midswing (MS). Each positive peak is accompanied by two negative peaks (or minima) on either side which indicate the reversal of leg velocity direction. The negative peak (NP) preceding the MS is identified as the TO event while the NP after the MS is marked as a HS.

The article "Estimation of Gait Parameters for Transfemoral Amputees Using Lower Limb Kinematics and Deterministic Algorithms" was published in 2022. Journal: Appl Bionics Biomech.

In addition, the ZC of the velocity in the same signal are also identified and marked as the potential predictors of gait events as proposed by some authors [10], [16]. These are termed S-ZC and F-ZC algorithms for shank and foot segments, respectively.

Lastly, a novel algorithm is developed which uses the thigh angular velocity signal as the input. The positive peaks in the signal are marked as the TO instants while the negative peaks right after the positive peaks are marked as HS (cf. Figure 1). This is referred to as T-MM (thigh min–max) algorithm in this article.

Velocity signal for a complete gait trial comprising of 12–15 gait cycles is fed to the algorithm. All algorithms begin by identifying the positive peaks in the signal. To discriminate between the valid and false peaks, only the peaks above a certain threshold are detected. This threshold is calculated by taking the absolute mean of all data points in the signal. Reference HS and TO events were identified using a 10 N threshold on the GRF data.

### 2.4. Statistical Analysis

For each walking cycle, the timings for the TO and HS events obtained by this algorithm were compared against the force platform-based timings as the reference. The errors (eTO and eHS) were calculated by taking the difference between the corresponding predicted and reference events.

(1) $$\begin{array}{c} \text{Error}\left(\text{eHS}/\text{eTO}\right)=t_{\text{reference}}-t_{\text{predicted}}, \end{array}$$

where the actual events refer to the ones marked using the force platform. The error is positive when the predicted event precedes the actual event and vice versa. A 5-number summary statistic (involving the median, lower and upper quartiles, minimum, and maximum values) was selected for further descriptive analysis. Descriptive statistics of mean error (ME) and mean absolute error (MAE) are also reported. Only complete gait cycles (defined as HS-HS for the same leg) were analyzed while the half-cycles at the start and end of the trials were discarded. Statistical tests of significance were performed at *p* = 0.05 level for group differences. Temporal gait parameters including step and stride times, stance, and swing phase durations were also computed. Results were exported to R statistical tool [37] for plotting and statistical testing.

The article "Estimation of Gait Parameters for Transfemoral Amputees Using Lower Limb Kinematics and Deterministic Algorithms" was published in 2022. Journal: Appl Bionics Biomech.

A variety of accuracy thresholds are used in the literature to accept or reject an algorithm ranging from 18 to 40 ms (e.g., [3] and [29]). To the best of the authors' knowledge, a universal criterion for the acceptance or rejection of an algorithm based on error magnitude does not exist. In this study, an accuracy threshold of ±25 ms on median error was set. When normalized, this threshold translates to <2.5% of the cycle/stride time at most walking speeds. Algorithms with greater errors than this band were considered inaccurate.

## 3. Results

TO and HS events for a total of 3398 walking cycles from 270 trials were compared. Results for the HS event from all algorithms are summarized in Figure 2(a). The DM algorithm on the shank velocity (S-DM) appeared to provide the best median estimate of HS (median error: −3 and −14 ms for sound and prosthetic sides, respectively). The DM algorithm based on foot velocity (F-DM) also provided reasonable accuracy for the HS event, though it provided a slightly larger-than-acceptable median error on the sound side (−27 ms). ZC algorithms as well as the thigh-based HS prediction provided inferior accuracy.

TO prediction results are shown in Figure 2(b). The median errors were larger than the threshold of ±25 ms for foot and shank-based methods. Only the thigh velocity algorithm provided the requisite accuracy with a median error of only 19 and −14 ms on sound and prosthetic sides, respectively.

The accompanying violin plots in Figure 2 show the distribution of error values. The plots did not present large skewness in most cases.

### 3.1. Mean Absolute Errors

Table 2 shows the MAE for both events from all five algorithms. The errors are further separated by leg side (sound vs. prosthetic).

For HS, the F-DM method produced the best result with an absolute ME of 18.2 ms (SD =12.9). The error was particularly low on the prosthetic side (~8 ms) and a small dispersion around the mean. S-DM algorithm also provided reasonable accuracy (~28 ms) and could be a potential candidate for HS prediction.

For the TO event, the T-MM gave an absolute error of ~35 ms. Moreover, it provided similar accuracy for both sound and prosthetic legs. The F-ZC algorithm based on foot velocity had a smaller overall error value (~30 ms) but it performed poorly on the prosthetic side with an absolute mean of ~48 ms.

### 3.2. Estimation of Gait Parameters

A key objective of gait event detection is to determine temporal gait parameters which depend upon the accuracy with which the events are detected in the first place. From the analysis of the above results, it can be deduced that no single algorithm can accurately predict both events, especially for both legs. This leads us to propose a hybrid approach that combines the strengths of multiple algorithms for the determination of gait parameters.

The article "Estimation of Gait Parameters for Transfemoral Amputees Using Lower Limb Kinematics and Deterministic Algorithms" was published in 2022. Journal: Appl Bionics Biomech.

Two combination algorithms are proposed in this regard. Both algorithms utilize the same TO prediction from the thigh-based T-MM algorithm due to its small error and robustness against the leg side. However, they differ in the HS prediction. In the first algorithm (termed hybrid shank–thigh or h-ST algorithm), the HS prediction from the S-DM method is used, while in the second hybrid algorithm, the HS prediction from F-DM is used (hence termed as h-FT algorithm). Box and whisker plots for errors in four gait parameters are plotted in Figure 3. Mean errors are also indicated by a circle. For comparison, errors from two traditional algorithms (S-DM and F-DM) are also plotted while the corresponding zero-crossing algorithms (S-ZC and F-ZC) are left out due to large HS median errors and several outliers especially on the prosthetic side (cf. Figure 2).

Stride and step times, which depend solely on the HS estimation, are estimated rather accurately by all algorithms. However, the hybrid h-ST and h-FT algorithms outperformed the traditional algorithms for the stance and double support time estimation. Of the two hybrid algorithms, the h-ST algorithm produced better results with median errors within ±25 ms range threshold in all cases.

The h-ST algorithm was further analyzed for its robustness against gait speed (0.4–1.4 m/s) and subjects' K-level.  Figure 4 summarizes the error results of the four gait parameters normalized by stride time. Median error values remained well within 5% of stride time for all gait parameters. Furthermore, correlation and Bland–Altman plots are also provided in the Appendix (see Figures 5 and 6).

## 4. Discussion and Conclusions

This study aimed at exploring different kinematic algorithms for the estimation of gait events and parameters for the amputee population. Among the velocity-based algorithm implemented, foot velocity provided the best estimate of the HS event, while a novel thigh velocity-based algorithm resulted in the best TO estimation. When combined, the hybrid h-ST algorithm provided the best results for key temporal gait parameters.

### 4.1. Accuracy of Gait Event Prediction

Prediction of gait events from kinematics has been a subject of many studies. Numerous studies have favored the shank-based DM method. While the literature agrees that this method is valid for HS prediction, recent studies have reported consistent early TO prediction [24]. Our results confirm this finding for the amputee population in this data set (cf.  Figure 3(b), panel labeled S-DM). On the other hand, some studies have advocated the use of ZC as a potential TO indicator [10], [16]. This proposition is not supported by our results as it resulted in the consistent late prediction (Figure 2, panel S-ZC). The same is true for the foot-based DM and ZC methods, albeit with smaller absolute error values (cf. Table 2). In this regard, a major contribution of this article is the presentation of the thigh-velocity-based T-MM algorithm for an improved TO estimation. The algorithm provided a similar median TO bias of (<20 ms) for both sound and prosthetic legs.

The article "Estimation of Gait Parameters for Transfemoral Amputees Using Lower Limb Kinematics and Deterministic Algorithms" was published in 2022. Journal: Appl Bionics Biomech.

On the other hand, the S-DM method provided the best accuracy for HS prediction confirming the findings of similar studies reporting errors in the range of 8–14 ms [6], [19]. Combining the HS estimation from the F-DM method and TO estimation from the T-MM algorithm greatly enhances the gait parameter accuracy as compared to single-limb-based estimation. This hybrid approach was also advocated in [3] yet is still unexplored. Moreover, as shown in Figure 4, the algorithm is robust against gait speed and subjects' K-level with a median error of less than 5% of stride time. An additional strength of this algorithm is the absence of any restrained time intervals for the events to occur. This results in a reduced computational cost during implementation. Moreover, the peak threshold (to discriminate between the actual peaks and the false peaks) is calculated automatically for each trial by taking the absolute mean of the input velocity signal eliminating the need for any manual adjustment for different speeds or subjects.

### 4.2. Limitations and Future Work

A key limitation of this study is the use of data acquired on a treadmill resulting in minimal gait variations. In a less constraining environment, the amputee gait could present a more varying gait making the prediction task more challenging. Moreover, to generalize the results, the algorithm should be validated on other populations with gait disorders, such as the patients suffering from Parkinson's disease.

## Figures and Tables

**Figure 1:** Representative thigh, shank, and foot angular velocity signals and the landmarks detected by the algorithms. The maxima/minima are indicated by a box (□) while the zero-crossings are indicated by a circle (○).

**Figure 2:** Plots of heel strike (a) and toe-off (b) errors for all five algorithms. The box indicates the lower and upper quartiles with the central line showing the median. The top and bottom lines of the box represent, respectively, the medians for the upper and lower halves of the data and the whiskers represent the highest and lowest values of the distribution, excluding outliers. Outliers are also presented as black dots. Boxplots are superimposed with violin plots (in grey) indicating error distribution. A hollow circle inside the box indicates the mean value. The plots are further separated by the leg side (sound vs. prosthetic). In addition, a green rectangle on each plot shows the acceptable median error range.

The article "Estimation of Gait Parameters for Transfemoral Amputees Using Lower Limb Kinematics and Deterministic Algorithms" was published in 2022. Journal: Appl Bionics Biomech.

**Figure 3:** Error plots of four gait parameters deduced from two conventional (panels 1 and 2) and two hybrid (panels 3 and 4) algorithms. The latter, with the inclusion of thigh-based TO estimation, result in improved prediction accuracy of the gait parameters. (Outliers are represented by dots, while mean value is indicated by a hollow circle).

**Figure 4:** Error plots for gait parameters using the h-ST algorithm. The x-axis shows the gait speed from 0.4 to 1.4 m/s while the y-axis represents error in terms of percentage of stride time. The blue dots indicate individual trial means.

**Figure 5:** Correlation and Bland–Altman plots for stance and double support time gait parameters calculated using the hybrid foot–thigh (h-ST) algorithm.

**Figure 6:** Correlation and Bland–Altman plots for step and stride time gait parameters calculated using the hybrid foot–thigh (h-ST) algorithm.

**Table 1:** List of subjects for whom the walking data are used in this study.

Subjects	Age	Gender	Mass (kg)	Height (m)	Etiology	Age of amputation (years)	K-level	Prescribed prosthesis		Number of trials
								Knee	Ankle	
TF01	26	Male	64.9	1.78	Traumatic	5	K3	Plie FI	AllPro FI	21
TF05	72	Male	79.4	1.65	Traumatic	4	K2	C-Leg Obk	Triton Low Profile Obk	25
TF07	49	Male	102.1	1.91	Traumatic	10	K3	C-Leg Obk	Triton Obk	22
TF08	42	Male	95.3	1.85	Traumatic	6	K3	Rheo Os	AllPro FI	25
TF09	65	Male	69.4	1.70	Traumatic	2	K2	C-Leg Obk	Trias Obk	25
TF11	51	Male	70.3	1.68	Traumatic	33	K3	C-Leg Obk	Trias Obk	23
TF12	59	Male	99.8	1.83	Traumatic	16	K2	C-Leg Obk	Trias Obk	23
TF13	61	Male	88.5	1.88	Traumatic	3	K3	Rheo Os	Proflex XC Os	20
TF15	23	Female	68.0	1.75	Traumatic	5	K3	Plie FI	Proflex XC Os	11
TF16	36	Male	100.2	1.80	Traumatic	8	K3	C-Leg Obk	AllPro FI	25
TF17	38	Male	104.3	1.91	Traumatic	33	K3	Plie FI	Soleus ClgPk	25
TF19	30	Female	59.0	1.60	Traumatic	10	K3	3R80 Obk	AllPro FI	25
Mean (SD)	46.0 (15.4)		83.4 (16.0)	1.8 (0.1)		11.3 (10.4)				

Complete details on amputation can be found in [34].

**Table 2:** Mean absolute error values for HS and TO from the five algorithms (CI: confidence interval).

Events	Algorithm	Mean absolute error (±SD) [95% CI]	Leg side	Mean absolute error (±SD)
Heel strike (HS)	T-MM	112.2 (±46.5)	Sound	85.67 (±16.0)
		[108.5, 115.2]	Prosthetic	138.60 (±51.6)
	S-DM	28.17 (±20.3)	Sound	16.72 (±13.5)
		[26.5, 29.8]	Prosthetic	39.61 (±19.4)
	S-ZC	49.25 (±32.9)	Sound	29.62 (±11.2)
		[47.1, 51.3]	Prosthetic	68.88 (±35.6)
	F-DM	18.27 (±12.9)	Sound	28.87 (9.5)
		[17.6, 19]	Prosthetic	7.68 (±4.2)
	F-ZC	48.25 (±33.4)	Sound	28.08 (±9.1)
		[47.3, 62.4]	Prosthetic	68.42 (±36.5)
Toe-off (TO)	T-MM	35.07 (±17.5)	Sound	36.22 (±15.4)
		[33.5, 36.4]	Prosthetic	33.92 (±19.3)
	S-DM	58.70 (±28.6)	Sound	82.05 (±20.8)
		[57.2, 60.2]	Prosthetic	35.36 (±10.7)
	S-ZC	40.86 (±14.5)	Sound	31.65 (±10.6)
		[39.8, 41.9]	Prosthetic	50.06 (±11.8)
	F-DM	45.96 (±9.3)	Sound	48.28 (±7.5)
		[42.2, 46.7]	Prosthetic	43.64 (±10.3)
	F-ZC	29.92 (±20.8)	Sound	11.63 (±6.6)
		[29.1, 30.7]	Prosthetic	48.21 (±12.3)

The article "Estimation of Gait Parameters for Transfemoral Amputees Using Lower Limb Kinematics and Deterministic Algorithms" was published in 2022. Journal: Appl Bionics Biomech.

## Data Availability

Data supporting this research article are available from the corresponding author or first author on reasonable request.

## Appendix

Correlation and Bland–Altman plots for four gait parameters calculated using the hybrid foot–thigh (h-ST) algorithm. All units are in milliseconds.
